# Treatment of Acute Pulmonary Embolism: Update on Newer Pharmacologic and Interventional Strategies

This article has been retracted.

**DOI:** 10.1155/2014/410341

**Published:** 2014-06-15

**Authors:** Francesco Pelliccia, Michele Schiariti, Claudio Terzano, Abdul M. Keylani, Darrin C. D'Agostino, Giuseppe Speziale, Cesare Greco, Carlo Gaudio

**Affiliations:** ^1^Department of Heart and Great Vessels “Attilio Reale”, Sapienza University, Viale del Policlinico 155, 00161 Rome, Italy; ^2^Respiratory Diseases Unit, “Sapienza” University, Rome, Italy; ^3^Department of Internal Medicine, Division of Cardiology, University of North Texas Health Science Center, Fort Worth, TX, USA; ^4^Anthea Hospital, GVM Care & Research, ES Health Science Foundation, Italy

## Abstract

Acute pulmonary embolism (PE) is a common complication in hospitalized patients, spanning multiple patient populations and crossing various therapeutic disciplines. Current treatment paradigm in patients with massive PE mandates prompt risk stratification with aggressive therapeutic strategies. With the advent of endovascular technologies, various catheter-based thrombectomy and thrombolytic devices are available to treat patients with massive or submassive PE. In this paper, a variety of newer treatment strategies for PE are analyzed, with special emphasis on various interventional treatment strategies. Clinical evidence for utilizing endovascular treatment modalities, based on our institutional experience as well as a literature review, is provided.

## 1. Introduction

Acute massive pulmonary embolism (PE) is a common life-threatening condition and represents the most serious manifestation along the spectrum of venous thromboembolic disease. In the United States, an estimated 530,000 cases of symptomatic PE occur annually [1], and approximately 300,000 people die every year from acute PE [2]. The mortality rate can exceed 58% in patients with acute PE presenting with hemodynamic shock [3], and most of these deaths occur within 1 hour of presentation [4]. Indeed, acute PE is believed to be the third most common cause of death among hospitalized patients [5], and, with an aging population, the number of people with PE is expected to increase.

The present paper reviews clinical risk assessment of PE as well as the efficacy and safety of the newer pharmacologic and catheter-directed (CDT) therapies.

## 2. Pathophysiology of Acute Pulmonary Embolism

To identify appropriate candidates for intensive treatment, physicians must be familiar with the clinical diagnosis of acute PE and understand the underlying pathophysiology. Life-threatening acute PE results whenever the combination of embolism size and underlying cardiopulmonary status interacts to produce hemodynamic instability [4]. The pathophysiology of PE consists of direct physical obstruction of the pulmonary arteries, hypoxemic vasoconstriction, and release of potent pulmonary arterial vasoconstrictors, which further increase pulmonary vascular resistance and right ventricular (RV) afterload. Acute RV pressure overload may result in RV hypokinesis and dilation, tricuspid regurgitation, and ultimately, RV failure.

## 3. Presenting Features of Acute Pulmonary Embolism

Patients with acute PE often present with dyspnea or chest pain, which may be sudden in onset or evolves over a period of days to weeks. If pulmonary infarction occurs, patients may also experience pleuritic chest pain with hemoptysis. Additionally, there are many nonspecific signs and symptoms including tachypnea, tachycardia, palpitations, light-headedness, fever, cough, wheezing, and rales. The possibility of massive PE should be considered in patients who have a sudden onset of near-syncope or syncope, hypotension, extreme hypoxemia, electromechanical dissociation, or cardiac arrest [2]. Some biomarkers may offer useful clinical information. Cardiac troponin levels may be elevated, particularly in patients with acute massive or submassive PE in whom clot burden is significant enough to overwhelm the patient's underlying cardiopulmonary reserve. Elevations in plasma B-type natriuretic peptide have been also been described in patients who have RV dysfunction from acute PE [6]. The d-dimer test measures plasma levels of a specific derivative of cross-linked fibrin to indicate possible presence of PE. The test has superior sensitivity (96%–98%) but must be interpreted together with clinical presentation because the test alone is nonspecific and may show a positive result in patients with cancer, infection, injury, and underlying inflammatory conditions. Of the various techniques of diagnostic imaging, CT angiography has the greatest sensitivity and specificity for detecting emboli in the main, lobar, or segmental pulmonary arteries. Systematic reviews and prospective randomized trials suggest that outpatients with suspected PE and negative CT angiographic studies have excellent outcomes without therapy [7]. The echocardiogram can be obtained at bedside, and the study may reveal findings that strongly support hemodynamically significant PE [8], offering the potential to guide treatment escalation to thrombolytic or endovascular therapy. Large emboli moving from the heart to the lungs are occasionally confirmed with this technique.

## 4. Indications for Advanced Therapy for Acute Pulmonary Embolism

In the 2008 publication by the American College of Chest Physicians,* Evidence-Based Clinical Practice Guidelines Regarding Treatment of PE*, therapeutic strategies of interventions, including thrombolysis and percutaneous embolectomy, were recommended based on appropriate risk stratification in highly selected patients who have PE-related hemodynamic instability [9]. A separate consensus guideline by the 2008 European Society of Cardiology Task Force regarding PE management shared many similar diagnostic criteria and therapeutic recommendations in patients with massive PE who experienced cardiogenic shock [10]. As regards risk stratification in patients with PE, scientific guidelines state that acute pulmonary embolism can be classified into three subtypes: massive, submassive, and stable [11].

- Massive pulmonary embolism is defined by hemodynamic instability (systolic blood pressure <90 mm Hg or decrease from baseline >40 mm Hg or cardiac arrest) and by symptom manifestation related to hypotension, tissue hypoperfusion, and hypoxemia.
- Submassive pulmonary embolism is when the patient is hemodynamically stable (systolic blood pressure ≥90 mm Hg) but with evidence of RV dysfunction as the direct, compensatory result of increased pulmonary artery pressures [12].
- Stable patients at low-risk are those who are normotensive with normal biomarker levels, no RV dysfunction on imaging, and short-term mortality rates approaching *≈*1%.

## 5. Medical Treatment of Acute Massive Pulmonary Embolism

There is no clinical controversy about the utility of thrombolysis in the management of a massive PE, which occurs in approximately 5% of patients [13]. Unless absolute contraindications preclude therapy after careful consideration, thrombolytics should be started in accordance with guidelines [9, 10]. The controversy for thrombolytic therapy indication is primarily centered on patients who are hemodynamically stable but demonstrate evidence of RV dysfunction (see the following list), which accounts for 31–64% of all patients with PE [14]. 

*Recommendations for Fibrinolysis for Acute PE (Adapted by [10])*

1. Fibrinolysis is reasonable for patients with massive acute PE and acceptable risk of bleeding complications* (Class IIa; Level of Evidence B).*
2. Fibrinolysis may be considered for patients with submassive acute PE judged to have clinical evidence of adverse prognosis (new hemodynamic instability, worsening respiratory insufficiency, severe RV dysfunction, or major myocardial necrosis) and low risk of bleeding complications* (Class IIb; Level of Evidence C).*
3. Fibrinolysis is not recommended for patients with low-risk PE* (Class III; Level of Evidence B)* or submassive acute PE with minor RV dysfunction, minor myocardial necrosis, and no clinical worsening* (Class III; Level of Evidence B).*
4. Fibrinolysis is not recommended for undifferentiated cardiac arrest* (Class III; Level of Evidence B).*

Thrombolytic agents activate plasminogen, which hydrolyzes a peptide bond and forms free plasmin. Only fibrin-bound plasmin is protected from the body's neutralizing enzyme, *α*-antiplasmin. Within a thrombus, plasmin hydrolyzes several key bonds, promoting clot lysis. In acute PE, thrombolysis has been shown to decrease pulmonary pressures within 2 hours of therapy. Although most benefits have been described if administered within 48 hours of symptom onset, enhanced clot lysis has been identified when thrombolytic therapy is administered up to 2 weeks after the onset of symptoms. Currently, only three thrombolytic agents have been approved by the United States Food and Drug Administration for the treatment of acute PE: streptokinase, urokinase, and alteplase. Nonselective agents, including urokinase and streptokinase, activate both circulating and clot-bound plasminogen. The practical uses of these agents are limited, as streptokinase has antigenic potential exacerbating hypotension, and urokinase in unconcentrated formulations intended for lysis of vascular lines, too low of a concentration in acute PE. Alteplase, however, is fibrin specific, binding preferentially to clot-bound plasminogen. Although fibrin-selective thrombolytic agents have not been evaluated for superior efficacy over nonselective agents for PE, if indicated, alteplase is often selected in clinical practice for the management of acute PE, due to its increased availability and more tolerable infusion reactions. In patients with acute PE, peripheral venous administration of thrombolytics is preferred. In high-risk patients unable to receive thrombolytic therapy or whose critical status does not allow sufficient time for systemic thrombolytic therapy to be effective, the use of interventional catheterization techniques should be considered.

## 6. Inferior Vena Cava Filters

Caval filters may be used as a means of primary or secondary PE prevention. Recent epidemiological data suggest that the combination of thrombolytic therapy with the placement of a vena cava filter may be particularly effective in lowering case fatality rates in unstable patients. At present, retrievable inferior vena cava filters have a place mostly when anticoagulation is absolutely contraindicated, or in cases of recurrence despite therapeutic dosing of anticoagulants [15].

## 7. Catheter-Directed Treatment of PE

### 7.1. Rationale for Catheter-Directed Treatment of Massive PE

Although alteplase is indicated for treatment of acute massive PE, many patients cannot receive systemic thrombolysis due to contraindications, and even when patients with acute PE are prescreened for absolute contraindications, the rate of major hemorrhage from systemic thrombolytic administration is approximately 20%, including a 3%–5% risk of hemorrhagic stroke [3]. Furthermore, there may be insufficient time in the acute setting to infuse full-dose thrombolytic agent. For these patients, CDT with no or low-dose local alteplase should be considered if available [9], and the decision should be made as part of a multidisciplinary discussion involving the interventionist and the patient's medical team. Specific indications for the use of CDT for acute PE have been published (see the following list) and should be used as guidelines to select candidates for endovascular therapy. The American College of Chest Physicians currently recommends that CDT be considered in selected highly compromised patients with PE who are unable to receive thrombolytic therapy because of bleeding risk [9] but global meta-analytic data have also demonstrated that CDT can be considered as a first-line treatment option in lieu of alteplase [16].

*Recommendations for Catheter-Derived Treatment of PE (Adapted by [10]) *

1. Depending on local expertise, either catheter embolectomy and fragmentation or surgical embolectomy is reasonable for patients with massive PE and contraindications to fibrinolysis* (Class IIa; Level of Evidence C)*.
2. Catheter embolectomy and fragmentation or surgical embolectomy is reasonable for patients with massive PE who remain unstable after receiving fibrinolysis* (Class IIa; Level of Evidence C)*.
3. For patients with massive PE who cannot receive fibrinolysis or who remain unstable after fibrinolysis, it is reasonable to consider transfer to an institution experienced in either catheter embolectomy or surgical embolectomy if these procedures are not available locally and safe transfer can be achieved* (Class IIa; Level of Evidence C)*.
4. Either catheter embolectomy or surgical embolectomy may be considered for patients with submassive acute PE judged to have clinical evidence of adverse prognosis (new hemodynamic instability, worsening respiratory failure, severe RV dysfunction, or major myocardial necrosis)* (Class IIb; Level of Evidence C)*.
5. Catheter embolectomy and surgical thrombectomy are not recommended for patients with low-risk PE or submassive acute PE with minor RV dysfunction, minor myocardial necrosis, and no clinical worsening* (Class III; Level of Evidence C).*

A variety of endovascular treatment strategies, including catheter-based thrombolysis and percutaneous pulmonary embolectomy, have been reported in the literature for patients with acute PE [2]. The reported mortality rates based on these various endovascular techniques vary from 0% to 25% [2]. Many of these percutaneous mechanical thrombectomy devices were used in conjunction with pharmacological thrombolysis, a technique also known as pharmacomechanical thrombectomy, which is a commonly adapted interventional technique in iliofemoral interventions [17]. Partly because of the heterogeneity of these endovascular treatment strategies, it is difficult to determine the most efficacious treatment strategy because no controlled trial is available. Nonetheless, brief overviews of these various treatment strategies are provided below.

### 7.2. Catheter-Directed Thrombolytic Therapy

The efficacy of CDT with intrapulmonary thrombolytic infusion in patients with acute massive PE has been reported in several studies with an overall remarkable treatment success [6]. This treatment strategy requires selective infusion catheter placement in the pulmonary artery within the embolus, followed by continuous infusion of thrombolytic drugs over a period of time. The treatment objective is to accelerate thrombus dissolution and achieve rapid reperfusion of the pulmonary arteries. In an ideal scenario, this catheter-directed intervention results in hemodynamic improvement with restoration of RV hypokinesis, normalization of RV size, and reduction of abnormally high pulmonary arterial pressures. Intrapulmonary administration of thrombolytic agents may potentially promote intravascular fibrinolysis elsewhere in the pelvis or lower extremity, thereby, reducing the likelihood of recurrent venous thromboembolism. Another therapeutic advantage of this intervention includes potential reduction of chronic elevations of pulmonary vascular resistance by improving pulmonary capillary blood flow, which might theoretically lower the incidence of long-term pulmonary hypertension.

Although CDT offers many theoretical benefits and therapeutic advantages in patients with PE, several major limitations must be acknowledged with this treatment approach. First, the risk of hemorrhagic complications, including intracranial or gastrointestinal bleeding, increases significantly with the treatment duration and thrombolytic dosage. This is a particular concern in elderly patients in whom catastrophic intracranial bleeding has been reported in clinical thrombolytic trials of arterial thrombosis [18]. Second, there has been only 1 single randomized trial, with only 8 patients, of whom 4 received streptokinase plus heparin and 4 received anticoagulation alone, which demonstrated survival advantage with thrombolytic therapy [19]. The survival benefit of CDT in PE remains to be proven in other clinical investigations. In contrast, findings from the ICOPER suggested that patients with massive PE treated with thrombolysis might not experience any survival advantage or reduction in major cardiovascular adverse events [3].

### 7.3. AngioJet Rheolytic Thrombectomy Catheter

The AngioJet Xpeedior thrombectomy device (Possis/Medrad; Minneapolis, MN) is a 6F over-the-wire catheter, which creates thrombus aspiration force based on Venturi's principle (Figure 1). The device permits a concomitant infusion of the thrombolytic agent, which creates a pharmacomechanical thrombectomy technique of thrombus dissolution by both thrombolysis and mechanical thrombectomy [20]. The pharmacomechanical thrombectomy technique using this device is widely used in deep venous thrombosis interventions. Short-acting, newer-generation fibrinolytic drugs, such as alteplase (10 to 20 mg), reteplase (2.5 to 5 U), or tenecteplase (5 to 10 mg), may be used for the pharmacomechanical thrombectomy approach. However, because the AngioJet Xpeedior is not designed to treat vessels greater than 12 mm in diameter, its therapeutic efficacy in the treatment of massive PE remains limited [21–23]. Procedural-related complications and deaths have been reported using this device in PE interventions, thus prompting FDA to issue a black-box warning on the device. Based on safety concerns, the AngioJet device should not be used as the initial treatment in patients with acute massive PE.

### 7.4. Personal Experience

A total of 33 patients (43 ± 13 years, 20 men) with acute PE and contraindications to thrombolytic therapy were treated with Angiojet at a single tertiary referral center, IN Rome, Italy. Acute massive pulmonary embolism was initially diagnosed by computed tomography and then confirmed by pulmonary angiography. Pulmonary thrombus location was evaluated prior to the procedure. Anemia was defined as a decrease in hematocrit level <39% for men and <36% for women. Renal failure was defined as oliguria (urine output < 500 mL over 24 hours) or an increase in creatinine (>25% over baseline or an overall increase by 1 g/dL). Catheter thrombectomy with Angiojet resulted in immediate angiographic improvement in 22/23 patients, with a rapid amelioration in functional class (from 3.3 ± 0.9 to 2.1 ± 0.7, *P* < 0.001) and an increase in oxygen saturation (from 71 ± 15 to 92 ± 17%, *P* < 0.001). Side effects during the procedure included transient heart block (1 patient), hypotension (3 patients), and bradycardia (5 patients). After the procedure, anemia was detected in 4 patients, while no patient had evidence of developed renal failure. The clinical improvement was maintained while in hospital and during a 6-month follow-up period, with a progressive decrease to normal of the peak systolic pulmonary pressure (from 65 ± 31 to 31 ± 19 mm Hg, *P* < 0.001). Our experience indicates that in patients with acute massive PE and contraindications to thrombolysis, catheter thrombectomy with Angiojet is an effective therapeutic option not associated with relevant and persistent side effects, including the risk of developing anemia and renal failure.

## 8. Conclusion

Rapid risk stratification by identifying patients with acute massive and acute submassive PE is essential in determining appropriate treatment escalation beyond anticoagulation. In the urgent clinical setting, the decision to escalate therapy should be made as part of a multidisciplinary discussion involving the interventionist and the primary medical team. For patients with less severe or submassive PE, the use of endovascular treatment in the form of local thrombolytic drug infusion appears to be a promising option for reducing acute and chronic complications from PE while avoiding the bleeding risks from full-dose systemic thrombolysis [24]. For patients in extremis from massive PE, emergent treatment escalation is necessary in the form of systemic thrombolysis, CDT, or combination therapy depending on the circumstance. If alteplase is contraindicated or there is insufficient time for full-dose administration, CDT may be the only viable treatment option [25]. Indeed, at experienced centers, the use of modern CDT has proven to be a life-saving treatment in patients dying from acute massive PE. It is therefore recommended that all interventionists understand the rationale for CDT and become familiar with initiating CDT as a life-saving endovascular procedure.

## Figures and Tables

**Figure 1:** Selective angiography of the left main pulmonary artery demonstrated a massive pulmonary embolism of the left pulmonary artery with contrast-filling defect in the left pulmonary parenchyma (a). Multiple aspirations with the AngioJet Xpeedior thrombectomy device (Possis/Medrad, Minneapolis, MN) were then performed (b). Catheter thrombectomy with Angiojet resulted in immediate angiographic improvement (c).

## References

[1] Heit JA, Cohen AT, Anderson AT (2005). Estimated annual number of incident and recurrent, non-fatal and fatal venous thromboembolism (VTE) events in the U.S.. *Blood*.

[2] Tapson VF (2008). Acute pulmonary embolism. *The New England Journal of Medicine*.

[3] Goldhaber SZ, Visani L, De Rosa M (1999). Acute pulmonary embolism: clinical outcomes in the International Cooperative Pulmonary Embolism Registry (ICOPER). *The Lancet*.

[4] Wood KE (2002). Major pulmonary embolism: review of a pathophysiologic approach to the golden hour of hemodynamically significant pulmonary embolism. *Chest*.

[5] Pulido T, Aranda A, Zevallos MA (2006). Pulmonary embolism as a cause of death in patients with heart disease: an autopsy study. *Chest*.

[6] Melanson SEF, Laposata M, Camargo CA (2006). Combination of D-dimer and amino-terminal pro-B-type natriuretic peptide testing for the evaluation of dyspneic patients with and without acute pulmonary embolism. *Archives of Pathology and Laboratory Medicine*.

[7] Moores LK, Jackson WL, Shorr AF, Jackson JL (2004). Meta-analysis: Outcomes in patients with suspected pulmonary embolism managed with computed tomographic pulmonary angiography. *Annals of Internal Medicine*.

[8] Goldhaber SZ, Haire WD, Feldstein ML (1993). Alteplase versus heparin in acute pulmonary embolism: randomised trial assessing right-ventricular function and pulmonary perfusion. *The Lancet*.

[9] Kearon C, Kahn SR, Agnelli G, Goldhaber S, Raskob GE, Comerota AJ (2008). Antithrombotic therapy for venous thromboembolic disease: American College of Chest Physicians evidence-based clinical practice guidelines (8th edition). *Chest*.

[10] Torbicki A, Perrier A, Konstantinides S (2008). Guidelines on the diagnosis and management of acute pulmonary embolism: the Task Force for the Diagnosis and Management of Acute Pulmonary Embolism of the European Society of Cardiology (ESC). *European Heart Journal*.

[11] Piazza G, Goldhaber SZ (2006). Acute pulmonary embolism. Part II: treatment and prophylaxis. *Circulation*.

[12] Ten Wolde M, Söhne M, Quak E, Mac Gillavry MR, Büller HR (2004). Prognostic value of echocardiographically assessed right ventricular dysfunction in patients with pulmonary embolism. *Archives of Internal Medicine*.

[13] Schoepf UJ, Kucher N, Kipfmueller F, Quiroz R, Costello P, Goldhaber SZ (2004). Right ventricular enlargement on chest computed tomography: a predictor of early death in acute pulmonary embolism. *Circulation*.

[14] Grifoni S, Olivotto I, Cecchini P (2000). Short-term clinical outcome of patients with acute pulmonary embolism, normal blood pressure, and echocardiographic right ventricular dysfunction. *Circulation*.

[15] Stein PD, Matta F, Keyes DC, Willyerd GL (2012). Impact of Vena Cava Filters on in-Hospital case fatality rate from pulmonary embolism. *The American Journal of Medicine*.

[16] Kuo WT, Gould MK, Louie JD, Rosenberg JK, Sze DY, Hofmann LV (2009). Catheter-directed therapy for the treatment of massive pulmonary embolism: systematic review and meta-analysis of modern techniques. *Journal of Vascular and Interventional Radiology*.

[17] Li J-J, Zhai R-Y, Dai D-K, Gao K, Wei B-J, Wang C (2006). Interventional mechanical thrombectomy procedure in treating acute massive pulmonary infarction. *Journal of Interventional Radiology*.

[18] Krajina A, Lojík M, Chovanec V (2007). Percutaneous mechanical fragmentation of emboli in the pulmonary artery. *Ceska Radiologie*.

[19] Kuo WT, Van den Bosch MAAJ, Hofmann LV, Louie JD, Kothary N, Sze DY (2008). Catheter-directed embolectomy, fragmentation, and thrombolysis for the treatment of massive pulmonary embolism after failure of systemic thrombolysis. *Chest*.

[20] Siablis D, Karnabatidis D, Katsanos K, Kagadis GC, Zabakis P, Hahalis G (2005). AngioJet rheolytic thrombectomy versus local intrapulmonary thrombolysis in massive pulmonary embolism: a retrospective data analysis. *Journal of Endovascular Therapy*.

[21] Kuo WT, Sze DY, Hofmann LV (2008). Catheter-directed intervention for acute pulmonary embolism: a shining saber. *Chest*.

[22] Kucher N, Windecker S, Banz Y (2005). Percutaneous catheter thrombectomy device for acute pulmonary embolism: in vitro and in vivo testing. *Radiology*.

[23] Kucher N, Goldhaber SZ (2005). Management of massive pulmonary embolism. *Circulation*.

[24] Kennedy RJ, Kenney HH, Dunfee BL (2013). Thrombus resolution and hemodynamic recovery using ultrasound-accelerated thrombolysis in acute pulmonary embolism. *Journal of Vascular and Interventional Radiology*.

[25] Wells PS, Forgie MA, Rodger MA (2014). Treatment of venous thromboembolism. *JAMA: Journal of the American Medical Association*.

